The article "Lopsided Blood‐Thinning Drug Increases the Risk of Internal Flow Choking Leading to Shock Wave Generation Causing Asymptomatic Cardiovascular Disease" was retracted in 2024. Reasons: unreliable results or conclusions; concerns about the data; concerns about the results or conclusions.

# Lopsided Blood‐Thinning Drug Increases the Risk of Internal Flow Choking Leading to Shock Wave Generation Causing Asymptomatic Cardiovascular Disease

**DOI:** 10.1002/gch2.202000076

**Published:** 2021-01-29

**Authors:** Valsalayam Raghavapanicker Sanal Kumar, Shiv Kumar Choudhary, Pradeep Kumar Radhakrishnan, Rajaghatta Sundararam Bharath, Nichith Chandrasekaran, Vigneshwaran Sankar, Ajith Sukumaran, Charlie Oommen

**Affiliations:** ^1^ Vikram Sarabhai Space Centre (SC CA No.6301/2013) Indian Space Research Organisation Thiruvananthapuram Kerala 695022 India; ^2^ National Centre for Combustion Research and Development Indian Institute of Science Bangalore Karnataka 560012 India; ^3^ Department of Aeronautical Engineering Kumaraguru College of Technology Coimbatore Tamil Nadu 641049 India; ^4^ Department of Cardiothoracic and Vascular Surgery All India Institute of Medical Sciences New Delhi 110029 India; ^5^ Chief Division of Cardiothoracic and Vascular Surgery GITAM University Visakhapatnam Andhra Pradesh 530045 India; ^6^ Department of Aerospace Engineering Indian Institute of Technology Kanpur Uttar Pradesh 208016 India

**Keywords:** acute‐heart failure, asymptomatic hemorrhage, BHCR, biofluid choking, BPR, Covid‐19, sanal flow choking

## Abstract

The discovery of Sanal flow choking in the cardiovascular‐system calls for multidisciplinary and global action to develop innovative treatments and to develop new drugs to negate the risk of asymptomatic‐cardiovascular‐diseases. Herein, it is shown that when blood‐pressure‐ratio (BPR) reaches the lower‐critical‐hemorrhage‐index (LCHI) internal‐flow‐choking and shock wave generation can occur in the cardiovascular‐system, with sudden expansion/divergence/vasospasm or bifurcation regions, without prejudice to the percutaneous‐coronary‐intervention (PCI). Analytical findings reveal that the relatively high and the low blood‐viscosity are cardiovascular‐risk factors. In vitro studies have shown that nitrogen, oxygen, and carbon dioxide gases are dominant in fresh blood samples of humans/guinea pigs at a temperature range of 98.6–104 F. An in silico study demonstrated the Sanal flow choking phenomenon leading to shock‐wave generation and pressure‐overshoot in the cardiovascular‐system. It has been established that disproportionate blood‐thinning treatment increases the risk of the internal‐flow‐choking due to the enhanced boundary‐layer‐blockage‐factor, resulting from an increase in flow‐turbulence level in the cardiovascular‐system, caused by an increase in Reynolds number as a consequence of low blood‐viscosity. The cardiovascular‐risk can be diminished by concurrently lessening the viscosity of biofluid/blood and flow‐turbulence by raising the thermal‐tolerance‐level in terms of blood‐heat‐capacity‐ratio (BHCR) and/or by decreasing the systolic‐to‐diastolic blood‐pressure‐ratio.

The article "Lopsided Blood‐Thinning Drug Increases the Risk of Internal Flow Choking Leading to Shock Wave Generation Causing Asymptomatic Cardiovascular Disease" was retracted in 2024. Reasons: unreliable results or conclusions; concerns about the data; concerns about the results or conclusions.

## Graphical abstract

It has been shown that at a critical systolic‐to‐diastolic blood‐pressure‐ratio, the internal‐flow‐choking (biofluid/Sanal‐flow‐choking) can occur anywhere in the cardiovascular‐system with or without a plaque or stent. The uneven usage of blood‐thinning drugs increases cardiovascular‐risk because low blood‐viscosity is a risk‐factor for internal‐flow‐choking causing the shock‐wave generation at a critical‐pressure‐ratio.

## 1 Introduction

Discovery of Sanal flow choking (PMCID: PMC7267099)^[^ ^1^ ^]^ in the cardiovascular system calls for multidisciplinary and global actions to recommend innovative treatments and to develop new drugs to negate the risk of flow choking leading to shock wave generation causing asymptomatic cardiovascular disease. Admittedly, heart failure (HF) is the cardiovascular epidemic of the 21st century.^[^ ^2^ ^]^ The ischemic heart disease or coronary heart disease (CHD) refers to atherosclerosis of the coronary arteries, where the deposit of plaques cause reduced blood flow and/or arterial blockage. Cardiovascular disease (CVD) refers to all types of diseases that affect the heart or blood vessels, including CHD. Although there has been significant advancement in the diagnosis, prognosis, treatment, and prevention of heart failure with reduced ejection fraction, the morbidity and mortality are still extensive. This is particularly true due to the Covid‐19 pandemic (www.escardio.org). An ejection fraction is a blood flow measurement in percentage (%), specifying how much blood the left ventricle pumps out with each contraction. An ejection fraction measurement under 40% may be an indication of heart failure or cardiomyopathy. An ejection fraction from 41%–49% may be considered as “borderline” cases having the history of stroke^[^ ^3^ ^]^ (memory effect). A normal heart's ejection fraction may be between 50%–70%. An ejection fraction value higher than 75% generally indicates hypertrophic cardiomyopathy (HCM), which could affect people of any age. HCM is reported as a cause of acute heart failure particularly in young people, including young athletes.^[^ ^3^, ^4^, ^5^ ^]^ It is important to note that though all these percentage demarcations of the ejection fraction are meaningful for the diagnosis it was not supported by any closed‐form analytical model for taking an authentic conclusion on the desirable blood flow percentage for forecasting the risk of acute‐heart‐failure (AHF) and furthering medical management in an individual subject. The European Society of Cardiology (ESC) reported (2020) that subjects with cardiovascular‐risk factors and proven CVD denote an exposed population when agonizing from the Covid‐19. ESC also added that subjects with cardiac injury in the perspective of Covid‐19 have an enhanced risk of illness and demise (www.escardio.org). In light of the discovery of Sanal flow choking in the cardiovascular system,^[^ ^1^ ^]^ the thermal tolerance of the Covid‐19 patients’ blood needs to be examined in terms of biofluid/blood heat capacity ratio (BHCR) for the risk assessment of the cardiovascular disease.^[^ ^1^, ^2^ ^]^

AHF is reported as the biggest killer globally over the centuries. Very frequently, fatal AHF happens without prior indications of coronary artery obstruction (angina). According to the world health organization (WHO),^[^ ^6^ ^]^ ischemic heart disease (IHD)^[^ ^7^ ^]^ and asymptomatic hemorrhage(AH)*/*stroke are the world's biggest killers. The truly popular consequence of management with the blood‐thinning‐drug, causing to lower blood viscosity is bleeding and very frequently asymptomatic hemorrhage and acute heart failure happens without any preceding symptoms. Milton Packer^[^ ^8^ ^]^ reported (2018) that acute heart failure is an event and not an illness and put forward a coherent claim for multidisciplinary research and a paradigm shift in thinking in the therapeutic drug development with a focus on the chemistry of drugs.^[^ ^8^, ^9^ ^]^ This is particularly inevitable at this juncture due to the Covid‐19 pandemic and associated cardiovascular risk. V. R. S. Kumar et al.^[^ ^1^, ^10^, ^11^, ^12^, ^13^, ^14^, ^15^ ^]^ discovered (2018) that such a transient episode leading to asymptomatic hemorrhage and acute heart failure is due to the Sanal flow choking (due to the boundary layer blockage (BLB) induced convergent‐divergent (CD) nozzle flow effect) and/or biofluid choking (due to the plaque induced CD nozzle flow effect or due to vasospasm) at a critical systolic‐to‐diastolic blood pressure ratio (BPR) (see **Figure** **1**a–h). Note that the critical blood‐pressure‐ratio (BPR) for internal flow choking (Biofluid/Sanal flow choking) in the cardiovascular system (CVS) is exclusively decided by the biofluid/blood‐heat‐capacity‐ratio (BHCR).^[^ ^1^ ^]^ The Sanal flow choking phenomenon is established as the fluid‐throat induced internal flow choking in the real world flows (continuum/non‐continuum) due to the compressible viscous flow effect.^[^ ^1^ ^]^ An internal flow choking due to blood viscosity variations and turbulence in CVS leads to cavitation, shock wave generation, and transient pressure‐spike.^[^ ^1^, ^10^ ^]^ Note that internal flow choking could happen in vasospasm, vasa vasorum, and/or nanoscale tubes too.^[^ ^1^ ^]^ When the pressure of the nanofluid/non‐continuum‐flows increases, average‐mean‐free‐path decreases and thus, the Knudsen number reduces leading to a no‐slip boundary condition with compressible viscous flow effect. The Sanal flow choking is a compressible viscous flow effect creating a physical situation of sonic‐fluid‐throat in the CVS at a critical systolic‐to‐diastolic blood pressure ratio (SBP/DBP), due to the BLB.^[^ ^1^, ^10^, ^11^ ^]^

**Figure 1:** Demonstrations of the different physical situations of internal flow choking (Biofluid/Sanal flow choking) at a critical blood‐pressure‐ratio (BPR) without prejudice to the Percutaneous Coronary Intervention (PCI) in the cardiovascular system.^[^ ^1^ ^]^ a) Physical situation of biofluid choking in an artery with plaque deposit similar to a CD nozzle flow passage; b) A partially blocked artery demonstrating the CD nozzle flow passage causing biofluid choking; c) An apparently blocked artery with plaque deposit but with nanoscale fluid flow through the CD nozzle flow passage causing nanoscale biofluid flow choking; d) A partially blocked artery with stent creating a situation of biofluid flow choking at a critical BPR due to CD nozzle shaped flow passage; e) Demonstrating the physical situation of the Sanal flow choking at the presence of a stent in an artery with bifurcation; f) Demonstrating the physical situation of the Sanal flow choking in a healthy subject having an artery with bifurcation; g) Demonstrating the possibilities of biofluid choking and the Sanal flow choking in an artery with plaque and collateral circulation; h) Demonstrating the possibilities of biofluid choking at a critical BPR due to vasospasm.

The article "Lopsided Blood‐Thinning Drug Increases the Risk of Internal Flow Choking Leading to Shock Wave Generation Causing Asymptomatic Cardiovascular Disease" was retracted in 2024. Reasons: unreliable results or conclusions; concerns about the data; concerns about the results or conclusions.

We discovered through theoretical studies that, at the creeping inflow conditions, the blood/biofluid flow in the circulatory system with the sudden expansion/divergent/vasospasm/expansion valves/bifurcation duct, with or without any plaque or stent, could predispose to supersonic flow condition leading to the shock wave generation and pressure‐overshoot due to the phenomenon of internal flow choking (Biofluid/Sanal‐flow‐choking (See Figure 1a–h) as the Central Illustration) at a critical BPR due to the effect of BLB or convergent‐divergent (CD) nozzle flow effect.^[^ ^1^, ^10^, ^11^, ^12^, ^13^, ^14^, ^15^ ^]^ The BLB factor depends on the Mach number, viscosity of biofluid/blood, BHCR, and the flow turbulence level.^[^ ^1^, ^10^, ^11^ ^]^ The Sanal‐flow‐choking^[^ ^1^ ^]^ could happen in any blood vessel without an iota of the symptom of plaque. Note that Equation (1), derived from the compressible flow theory,^[^ ^11^ ^]^ is a condition set for prohibiting the internal‐flow‐choking in the circulatory system, which is defined herein as the hemorrhage index (HI). The HI highlights (see Equation (1)) the individual and group influences of biofluid dynamics, ejection fraction in terms of biofluid/blood flow rate (BFR), vessel geometry, specific heat of blood/biofluid at constant pressure (*C*_p_) and the other thermo‐physical properties of blood at the risk of internal flow choking leading to asymptomatic hemorrhage and acute heart failure.^[^ ^1^, ^10^, ^11^, ^12^, ^13^, ^14^, ^15^ ^]^

(1) $$\begin{array}{c} \begin{array}{l} HI=\frac{\text{Blood}\;\text{or}\;\text{Biofluid}\;\text{flow}\;\text{rate}}{\text{Vessel}\;\text{cross}\;\mathrm{sectional}\;\text{area}}\;\\ \sqrt{\frac{\left(\text{Prandtl}\;\text{Number}\right)\;\left(\text{Thermal}\;\text{Conductivity}\right)}{\left(\text{BHCR}\right)\;\left(\text{Density}\right)\;\left(C_{p}\right)\;\left(\text{Dynamic}\;\mathrm{Viscosity}\right)\;\left(\text{DBP}\right)}}\;<1 \end{array} \end{array}$$

(2) $$\begin{array}{c} LCHI={\left(\frac{{\left(BHCR\right)}_{\begin{array}{c} evolved\;gases\\ with\;the\;lowest\;BHCR \end{array}}+1}{2}\right)}^{{\left(BHCR\right)}_{lowest}/{\left(BHCR\right)}_{lowest}-1} \end{array}$$

(2a) $$\begin{array}{c} BPR=\frac{SBP}{DBP}<LCHI \end{array}$$

(3) $$\begin{array}{c} UCHI={\left(\frac{{\left(BHCR\right)}_{blood}+1}{2}\right)}^{{\left(BHCR\right)}_{blood}/{\left(BHCR\right)}_{blood}-1} \end{array}$$

Note that for prohibiting the spontaneous coronary artery dissection (SCAD) an unchoked‐fluid‐flow condition (HI < 1) must be satisfied throughout the circulatory system. It could be achieved by maintaining hemorrhage index (HI) always lower than one or the BPR always lower than the lower‐critical‐hemorrhage‐index (LCHI), which is dictated by the lowest value of the BHCR of evolved gases in the cardiovascular‐system (see Equation (2)). For instance, if carbon dioxide is the dominant gas in the cardiovascular‐system it is mandatory to maintain systolic‐to‐diastolic BPR lower than 1.8257 for creating an unchoked flow condition for prohibiting the shock wave generation^[^ ^1^ ^]^ causing the asymptomatic hemorrhage and acute heart failure. Equation (2) shows that the BHCR has a bearing on all the parameters highlighted in Equation (1) for prohibiting internal flow choking anywhere in the cardiovascular system. The fact is that at the choked flow condition the critical‐BPR is a unique function of BHCR. Note that Equations (1) and (2) are two independent analytical models highlighting the same physical situation and therefore both equations complement each other. It is evident from Equations (1) and (2a) that a decrease in diastolic blood pressure (DBP) increases cardiovascular risk, which correlates with existing clinical findings.^[^ ^1^, ^2^, ^3^, ^4^, ^5^, ^6^, ^7^, ^8^, ^9^, ^10^, ^11^, ^12^, ^13^, ^14^, ^15^, ^16^, ^17^, ^18^, ^19^, ^20^, ^21^, ^22^, ^23^, ^24^, ^25^, ^26^, ^27^, ^28^, ^29^, ^30^, ^31^, ^32^, ^33^, ^34^, ^35^, ^36^, ^37^, ^38^, ^39^, ^40^, ^41^, ^42^, ^43^, ^44^, ^45^, ^46^, ^47^, ^48^, ^49^, ^50^, ^51^, ^52^, ^53^, ^54^, ^55^, ^56^, ^57^, ^58^, ^59^, ^60^, ^61^, ^62^, ^63^, ^64^, ^65^, ^66^, ^67^, ^68^, ^69^, ^70^, ^71^, ^72^, ^73^, ^74^, ^75^, ^76^, ^77^, ^78^, ^79^, ^80^, ^81^, ^82^, ^83^ ^]^ Equation (2a) also reveals that an increase in systolic blood pressure (SBP) increases cardiovascular risk. In brief, an increase in BPR increases the cardiovascular risk.

The article "Lopsided Blood‐Thinning Drug Increases the Risk of Internal Flow Choking Leading to Shock Wave Generation Causing Asymptomatic Cardiovascular Disease" was retracted in 2024. Reasons: unreliable results or conclusions; concerns about the data; concerns about the results or conclusions.

The LCHI is predicted (see Equation (2)) using the lowest value of the BHCR among the dominant gases evolved from the blood samples of each subject (human being or animal). The upper critical hemorrhage index (UCHI) is predicted (see Equation (3)) from the specific heat of blood at constant pressure (*C*_p_) and the specific heat of blood at constant volume (*C*_v_), estimated using the Differential Scanning Calorimeter – Perkin Elmer DSC 8000.

Traditionally hypertension is considered as a cardiovascular risk factor in patients with systemic autoimmune and chronic inflammatory diseases. Until the dissemination of this article and connected articles^[^ ^1^, ^10^, ^11^, ^12^, ^13^, ^14^, ^15^, ^79^, ^80^, ^81^, ^82^, ^83^ ^]^ there were no authentic conclusions to support whether hypertension or hypotension is of more risk with regards to asymptomatic hemorrhage and acute heart failure.^[^ ^10^, ^11^, ^12^, ^13^, ^14^, ^15^, ^16^, ^17^, ^18^ ^]^ V. R. S. Kumar et al.^[^ ^1^, ^10^, ^11^, ^12^, ^13^, ^14^, ^15^ ^]^ reported that an AHF could occur in both hypertension or hypotension patients because the controlling parameter of this event is the BPR. In brief, attaining a critical BPR is considered as a risk factor for asymptomatic hemorrhage and acute heart failure. Therefore, at the threshold of the internal flow choking condition, a minor oscillation in BPR for both hyper and hypo subjects is likely to aggravate the risk of heart failure. In light of the discovery of flow choking in blood vessels, the classic definition of the hypertension causing cardiovascular risk is largely arbitrary (SBP ≥140 and/or DBP ≥90 mmHg). The prevailing cardiovascular risk data remains challenging owing to the fact that internal flow choking could occur in both hypertension or hypotension subjects once BPR reaches LCHI (see Equation (2a)). The Sanal flow choking could be negated by controlling the blood viscosity and turbulence altogether and/or by reducing BPR. Traditionally, blood viscosity is reduced by blood thinners. It is important to note that while decreasing the blood viscosity the Reynolds number will increase and the flow becomes turbulent, which increases the BLB factor causing an early Sanal flow choking. It implies that relatively high blood viscosity and low blood viscosity are risk factors of asymptomatic hemorrhage and acute heart failure.

The article "Lopsided Blood‐Thinning Drug Increases the Risk of Internal Flow Choking Leading to Shock Wave Generation Causing Asymptomatic Cardiovascular Disease" was retracted in 2024. Reasons: unreliable results or conclusions; concerns about the data; concerns about the results or conclusions.

There are two main types of blood thinners namely, anticoagulants such as heparin or warfarin and antiplatelet drugs, such as aspirin to prevent blood cells from clumping together to form a clot. According to a focused update^[^ ^19^ ^]^ and guidelines of the American Heart Association (AHA)/ACC/HRS, a new generation blood‐thinning drug, non‐vitamin K oral anticoagulants (NOACs), is now suggested as the favored substitute to warfarin for reducing the risk of stroke allied with atrial fibrillation (AFib). Note that large swings in BPR create periodic choking and unchoking phenomena causing atrial fibrillation or an irregular heartbeat (arrhythmia). This multidisciplinary review paper aims to highlight the fundamental cause(s) of asymptomatic cardiovascular disease and propose possible solutions for reducing the risk of asymptomatic hemorrhage and acute heart failure.

International normalized ratio (INR) is the chosen trial of option for subjects taking vitamin K antagonists (VKA), which helps to predict the risk of bleeding or the coagulation status of the subjects. Subjects using oral anticoagulants are essential to monitor INR to regulate the VKA quantities because these differ among subjects.^[^ ^20^ ^]^ The use of antiplatelet is frequently in grouping or as a substitute to anticoagulant. INR is utilized to decide the coagulation trend of blood and is necessary for blood thinning medication (especially warfarin). In general, for a healthy person the estimated normal range of INR is about one and it is reported that the INR is from 2.0 to 3.5 for subjects under anticoagulant therapy.^[^ ^21^ ^]^ An enhanced INR implies a high tendency of bleeding, whereas the lower INR is a warning of the high risk of having a thrombotic event in patients who are on anticoagulant therapy. Accordingly, anticoagulant and antiplatelet are exercised interchangeably, there is a conventional laboratory index, namely, INR for regular checking to assess contraindication to and/or need for anticoagulant; but none for antiplatelet.^[^ ^21^ ^]^ Therefore, this issue is worth addressing in terms of variations in whole blood viscosity and the altered turbulence level due to the blood thinning medication and/or seasonal effects. Note that the analytical prediction of the Sanal flow choking^[^ ^1^, ^10^, ^11^, ^12^, ^13^, ^14^, ^15^ ^]^ is a breakthrough in biological science, which creates a radical change in the diagnostic sciences of asymptomatic vascular diseases because the various causes of the Sanal flow choking are complementary with all the established concepts in medical sciences.^[^ ^1^, ^2^, ^3^, ^4^, ^5^, ^6^, ^7^, ^8^, ^9^, ^10^, ^11^, ^12^, ^13^, ^14^, ^15^, ^16^, ^17^, ^18^, ^19^, ^20^, ^21^, ^22^, ^23^, ^24^, ^25^, ^26^, ^27^, ^28^, ^29^, ^30^, ^31^, ^32^, ^33^, ^34^, ^35^, ^36^, ^37^, ^38^, ^39^, ^40^, ^41^, ^42^, ^43^, ^44^, ^45^, ^46^, ^47^, ^48^, ^49^, ^50^, ^51^, ^52^, ^53^, ^54^, ^55^, ^56^, ^57^, ^58^, ^59^, ^60^, ^61^, ^62^, ^63^, ^64^, ^65^, ^66^, ^67^, ^68^, ^69^, ^70^, ^71^, ^72^, ^73^, ^74^, ^75^, ^76^, ^77^, ^78^, ^79^, ^80^, ^81^, ^82^, ^83^ ^]^ The concepts of Sanal flow choking is well correlated herein with the existing theories and concepts in the biological sciences for finding possible solutions for reducing the risk of internal flow choking leading to shock wave generation causing the asymptomatic hemorrhage and acute heart failure.

The article "Lopsided Blood‐Thinning Drug Increases the Risk of Internal Flow Choking Leading to Shock Wave Generation Causing Asymptomatic Cardiovascular Disease" was retracted in 2024. Reasons: unreliable results or conclusions; concerns about the data; concerns about the results or conclusions.

Admittedly, whole blood viscosity is popularly the one of Virchow's triad, which is a recognized concept that pronounces the three widely found types of causes that are believed to interpose to thrombosis causing cardiovascular complications, namely, hypercoagulability, hemodynamic changes (stasis, turbulence), and endothelial injury/dysfunction. Further, it is well known that blood is a non‐Newtonian fluid^[^ ^22^, ^23^ ^]^ as blood viscosity changes due to fluid force and blood thinning medications. Viscosity variations are dependent on the shear rate or shear rate history of the blood/biofluid, which could vary due to seasonal effects too. Blood temperature decreases during the winter season resulting in an increase in blood viscosity and the inverse effect happens during the summer season.^[^ ^10^ ^]^ It corroborates that the BLB factor causing the Sanal flow choking would alter due to the blood viscosity variations as a consequence of the blood‐thinning medication and/or the seasonal effects.^[^ ^10^ ^]^ Indeed, BLB induced internal flow choking is more prone during the winter season than the summer season due to the higher blood viscosity at the relatively low blood temperature. It leads us to say that the risks of biofluid choking leading to asymptomatic hemorrhage and acute heart failure would be high during the winter than in the summer season, which is corroborating with the literature data.^[^ ^10^, ^17^ ^]^ It is important to note that blood‐thinning medication will increase the Reynolds number, which produces a high turbulence level creating an enhanced BLB factor causing an early flow choking. All these deliberations lead to corroborate that relatively high blood viscosity and low blood viscosity are risk factors for an early internal flow choking in cardiovascular system (CVS) causing asymptomatic stroke/hemorrhage and acute heart failure, which correlates with the established index, namely, the INR. Therefore, the real effect of viscosity on internal flow choking in CVS needs to be established to take preventive strategies for reducing the risk of asymptomatic hemorrhage and acute heart failure. On this rationale, it is essential, rather needed, perhaps inevitable to declare a condition for prohibiting the internal flow choking in the CVS, in terms of viscosity, density, Reynolds number, BHCR, BPR, ejection fraction, and stenosis (vessel geometry), which we have attempted herein through the closed‐form analytical methodology.

The article "Lopsided Blood‐Thinning Drug Increases the Risk of Internal Flow Choking Leading to Shock Wave Generation Causing Asymptomatic Cardiovascular Disease" was retracted in 2024. Reasons: unreliable results or conclusions; concerns about the data; concerns about the results or conclusions.

Rongjia Tao^[^ ^24^, ^25^ ^]^ narrated that decreasing the blood viscosity and concurrently reducing the turbulence level are the crucial missions to prevent acute heart failure. As stated earlier these two missions conflict with each other. Rongjia Tao^[^ ^24^ ^]^ further reported that the only recognized technique to decrease the blood viscosity is to take a drug, such as aspirin. Note that using medicine to reduce the blood viscosity only makes the turbulence worse and increases the chances of cavitation and biofluid choking because the BLB factor will be more for the turbulent flow than the laminar flow. The flow turbulence increases the deficit of energy in the form of friction, which increases the BLB in blood vessels and generates heat and augments the internal energy causing a decrease in the heat‐capacity‐ratio of blood/biofluid, which is vulnerable to an early flow choking in the cardiovascular system. Based on the above findings we established herein that the lopsided blood‐thinning drugs increase the risk of internal flow choking triggering acute heart failure, which supports the established laboratory index, namely, the INR. More specifically, an overdose of drugs for blood‐thinning medication increases the Reynolds number leading to the high turbulence level in the vessel and as a result the laminar flow could be disturbed and becomes turbulent causing an early internal flow choking causing a transient sharp pressure‐spike due to the generation of shock waves at the creeping inflow condition without any iota of symptoms of the plaque in an artery with sudden expansion/divergence/vasospasm/bifurcation (see Figure 1 as the Central Illustration). More precisely, internal flow choking could occur in vasa vasorum, nanoscale tubes, and also in the coronary artery without prejudice to the Percutaneous Coronary Intervention (PCI). Briefly, the prediction of internal flow choking in cardiovascular‐system is a scientific breakthrough and a paradigm shift in the diagnostic science of asymptomatic cardiovascular diseases. Sanal flow choking leads to the shock‐wave generation followed by pressure overshoot causing the tearing of the blood vessels. The tearing depends on the memory effects (stroke history) and the thermoviscoelastic properties of the vessel. This basic interdisciplinary research review paper, which originated from chemical rocket science,^[^ ^1^, ^10^, ^39^, ^59^ ^]^ aims to discover the fundamental cause(s) of bleeding while taking blood‐thinning drugs and propose possible solutions for reducing the risk of internal flow choking causing asymptomatic hemorrhage and acute heart failure. In a nutshell, the proof of the concept of Sanal flow choking in cardiovascular‐system leading to asymptomatic hemorrhage and acute heart failure is established herein through closed‐form analytical methodology, in vitro study and in silico modeling, which are briefly reviewed in the subsequent sections.

The article "Lopsided Blood‐Thinning Drug Increases the Risk of Internal Flow Choking Leading to Shock Wave Generation Causing Asymptomatic Cardiovascular Disease" was retracted in 2024. Reasons: unreliable results or conclusions; concerns about the data; concerns about the results or conclusions.

## 2 Analytical Methodology

The BLB in the blood vessels can be influenced by the variations in the blood viscosity and the BHCR of the flowing gas/nano plasma. The Equation (4) correlates the hydraulic diameter of the artery or any blood vessel (*d*_i_), the corresponding inflow Mach number (*M*), the axial Mach number (*M*_axial_), and the BHCR, which is derived from compressible flow theory.^[^ ^1^, ^11^ ^]^

(4) $$\begin{array}{c} BLB=\left[1-{\left[\frac{M_{inlet}}{M_{axis}}\right]}^{1/2}{\left[\frac{1+\left(\frac{BHCR-1}{2}\right)M_{axis}^{2}}{1+\left(\frac{BHCR-1}{2}\right)M_{inlet}^{2}}\right]}^{\frac{BHCR+1}{4\left(BHCR-1\right)}}\right]d_{i} \end{array}$$

The previous researchers, in general, assumed that the human blood is an incompressible fluid (i.e., C_p_ = C_v_). That is patently not true as the human blood specific volume (or density) does change with temperature or pressure. At the Sanal‐flow‐choking condition, the creeping flow will get accelerated in a uniform cross‐sectional area duct due to the area blockage caused by the boundary‐layer‐displacement‐thickness (i.e., the blockage factor, BLB). The 3D BLB at the Sanal‐flow‐choking condition (*M*_axis_ = 1) for diabatic flows (i.e., flow involves transfer of heat) is given in Equation (4a),^[^ ^1^, ^11^ ^]^

(4a) $$BLB|{}_{@sonic-fluid-throat}=\left[1-M_{inlet}^{1/2}{\left[\frac{2}{{\left(BHCR\right)}_{lowest}+1}\;\left(1\;+\;\frac{{\left(BHCR\right)}_{lowest}-1}{2}M_{inlet}^{2}\right)\right]}^{\;\frac{{\left(BHCR\right)}_{lowest}+1}{4\left(1-{\left(BHCR\right)}_{lowest}\right)}}\right]d_{i}$$

(5) $$\begin{array}{c} Mach\;Number<1 \end{array}$$

(5a) $$\begin{array}{c} V_{local}\sqrt{\frac{\left(Biofluid\;Density\right)}{\left(BHCR\right)\;\left(DBP\right)}}<1 \end{array}$$

(5b) $$\begin{array}{c} V_{local}\sqrt{\frac{C_{v}\left(Biofluid\;Density\right)}{C_{p}\left(DBP\right)}}<1 \end{array}$$

(5c) $$\begin{array}{c} {\left[\frac{{\left(BFR\right)}_{local}\;V_{local}}{{\left(BHCR\right)}_{lowest}\;\left(DBP\right)A_{local}}\right]}^{1/2}<1 \end{array}$$

(5d) $$\begin{array}{c} \begin{array}{l} \frac{\left(\text{Reynolds}\;\text{number}\right)\left(\text{kinematic}\;\mathrm{viscosity}\right)}{\text{Hydraulic}\;\text{diameter}\;\text{of}\;\text{the}\;\text{vessel}}\\ {\left[\frac{Blood\;Density}{\left(BHCR\right)\;\left(DBP\right)}\right]}^{1/2}<1 \end{array} \end{array}$$

The blockage factor in the blood vessels could change due to the seasonal effects as a consequence of the differences in blood viscosity.^[^ ^16^, ^17^, ^18^ ^]^ If the blood vessel geometry is similar to the convergent‐divergent (CD) nozzle shape or vasospasm (see Figure 1a–h)), the Sanal‐flow‐choking leads to shock wave generation and pressure‐overshoot.^[^ ^1^, ^10^, ^11^, ^12^, ^13^, ^14^, ^15^ ^]^ This physical situation can be predicted through the credible multidisciplinary in silico models,^[^ ^10^, ^11^, ^39^ ^]^ which must be verified and validated at the Sanal‐flow‐choking condition. **Figure** **2** shows (solution of Equation (4a)) the SANAL chart pertaining to a case of gas embolism with carbon dioxide as the dominant gas. It clearly indicates that irrespective of the percentage blockage of the artery, the critical BPR determines the risk of the internal‐flow‐choking leading to asymptomatic hemorrhage and acute heart failure. The SANAL chart also shows that a decrease in the blockage factor reduces the flow Mach number for meeting the continuity condition conceived from the law of nature, which reduces the risk of internal flow choking. Note that for prohibiting the internal flow choking all subjects (human being/animals) must maintain their systolic‐to‐diastolic BPR always lower than the LCHI (see Equations (2) and (2a)). Please note that BLB factor will never be zero in any real world flow system.^[^ ^1^, ^10^, ^11^ ^]^ Our analytical model proves that the stents could reduce the risk of the heart attack but no better than drugs owing to the fact that the Sanal flow choking could occur with and without stent (see Figure 1d–f)). Note that Equation (5) shows the condition for prohibiting the internal flow choking by maintaining Mach number (*M*) always less than one in the cardiovascular‐system. Mach number depends on the local velocity (*V*_local_) and local velocity of sound. Equations (5a)–(5c) are the corollary of Equation (5), which are derived from the compressible flow theory. It highlights various influencing parameters in prohibiting internal‐flow‐choking in an artery. Note that the ejection fraction is reflected in Equation (5c) in terms of BFR. It is evident from the closed‐form‐analytical model (see Equation (5c)) that the ejection fraction is not the lone parameter for declaring the risk of heart failure. It is coupled with the local vessel cross‐sectional area (*A*_local_), local velocity (*V*_local_), (BHCR)_lowest_, and the DBP. In high risk subjects (BPR close to LCHI or hemorrhage index close to 1.0) a minor swing in the BPR predisposes to the choking and the unchoking phenomena leading to arrhythmia. Most heart valve problems involve the aortic and mitral valves, possibly because of its geometric shape similar to a convergent‐divergent (CD) duct flow passage. Note that the internal‐flow‐choking could create unusual pressure‐overshoot in vessels with vasospasm, divergent/bifurcation regions, which increases memory effects (stroke history) leading to aneurysm and/or artery tear in the subsequent stroke.

The article "Lopsided Blood‐Thinning Drug Increases the Risk of Internal Flow Choking Leading to Shock Wave Generation Causing Asymptomatic Cardiovascular Disease" was retracted in 2024. Reasons: unreliable results or conclusions; concerns about the data; concerns about the results or conclusions.

**Figure 2:** SANAL Chart: Condition for prohibiting asymptomatic hemorrhage and acute heart failure (Solution curve of Equation (4a)).

It is abundantly clear from the physiological literature that the arterial wall material is viscoelastic and a priori knowledge of memory effects of such viscoelastic materials at multi‐axial stress conditions during the seasonal changes is necessary for understanding the behavior of the arterial tree better.^[^ ^42^, ^43^, ^44^, ^45^, ^46^, ^47^, ^48^, ^49^, ^50^, ^51^, ^52^, ^53^ ^]^ This is particularly true and inevitable for predicting the aneurysm and hemorrhagic‐stroke when the propagation of waves through such arteries, with diabatic flows (flow involves transfer of heat), having the vessel‐walls with thermoviscoelastic properties.^[^ ^42^, ^43^, ^59^ ^]^ Interestingly, the “memory effect,” (i.e., stress/stroke history herein) is the prominent characteristic of any viscoelastic material.^[^ ^59^ ^]^ Herein, we defined the memory effect as the stroke history wherein the current state of stress and past stroke histories determine the mechanical response of the material, namely, the onsite relaxation modulus of the blood vessels including vasa vasorum and capillaries. Therefore, an accurate and a priori knowledge of the combined effect of the rheology of biofluid and the thermoviscoelastic response of the vessels is inevitable for predicting an aneurysm and other asymptomatic cardiovascular diseases using the fluid‐structural interactive code calibrated with the credible Sanal flow choking condition.^[^ ^1^, ^10^, ^39^, ^79^ ^]^ For establishing the proof of the concept, we have demonstrated herein the Sanal flow choking and shockwave generation at a critical pressure ratio in a viscoelastic tube with vasospasm using air as the working fluid at the atmospheric exit flow condition (see Movie S1, Supporting Information). Further discussion of valve problems, aneurysm, and arrhythmia is beyond the scope of this review article.

The article "Lopsided Blood‐Thinning Drug Increases the Risk of Internal Flow Choking Leading to Shock Wave Generation Causing Asymptomatic Cardiovascular Disease" was retracted in 2024. Reasons: unreliable results or conclusions; concerns about the data; concerns about the results or conclusions.

## 3 In Vitro Methodology

We have estimated the BHCR, obtained from the blood samples of healthy human beings and a healthy Guinea pig living in the southern part of the Indian union, using the Differential Scanning Calorimeter (DSC) – Perkin Elmer DSC 8000. Please note that the ethical approval is not required by the national legislation of Indian union for conducting the blood sample test of healthy subjects. **Table** **1** shows the estimated UCHI of healthy human beings of ages 23–56 years. **Figure** **3** demonstrates the percentage variations of evolved gases (viz., N_2_ −m/z = 28, O_2_ −m/z = 32, CO_2_ −m/z = 44, Ar −m/z = 40, an unknown composite gas(CG) −m/z = 28.5), from the blood samples of four different healthy human beings and one healthy male Guinea pig four weeks old, during the hyphenated technique at a blood temperature of 40 °C (104 F). **Figure** **4** shows the mass spectrum of carbon dioxide (CO_2_) gas evolved as a function of both time and temperature obtained from blood sample tests of healthy subjects (human beings and a Guinea pig). We used a quadrupole mass spectrometer of Perkin Elmer make SQ8T with Electron Multiplier as the detector. During our comprehensive in vitro studies, we have noticed that the gases evolved from the fresh blood sample depends on the blood temperature, heating rate, blood group, age, and the blood pressure (BP) value. It is evident from Figures 3 and 4 that CO_2_ is consistently the dominant gas for human beings at a large temperature range whereas nitrogen (N_2_) gas is dominant in the blood sample of the Guinea pig.^[^ ^1^, ^14^, ^79^ ^]^ In light of Figure 4, the estimated lower critical hemorrhage index (LCHI) of all healthy human beings are found to be 1.8257, which is based on the evolved dominant carbon dioxide gas (BHCR = 1.289). In the case of Guinea pig, the LCHI is estimated as 1.8929, which is based on the dominant nitrogen (N_2_) gas (BHCR = 1.4) generated within the thermal tolerance level. We found that there are variations in the heat capacity of blood samples collected in three different Vacutainers of the same subjects. We have noticed that the anticoagulant reduces the BHCR and is susceptible to an early internal flow choking in blood vessels, including vasa vasorum, causing a high risk of asymptomatic hemorrhage, and acute heart failure. It is well known that the most common side effect of treatment with anticoagulant medicine is bleeding. Therefore, until the discovery of new drugs for increasing the BHCR, the physician should calculate and prescribe the doses of anticoagulant drug for each and every patient based on the clinical data of the individual subjects using the closed‐form analytical models presented herein (Equations (1), (2) and (5a)–(5c)) for prohibiting the internal flow choking causing asymptomatic hemorrhage and acute heart failure.

The article "Lopsided Blood‐Thinning Drug Increases the Risk of Internal Flow Choking Leading to Shock Wave Generation Causing Asymptomatic Cardiovascular Disease" was retracted in 2024. Reasons: unreliable results or conclusions; concerns about the data; concerns about the results or conclusions.

**Table 1:** Prediction of the UCHI from the heat capacity ratio of fresh blood samples of healthy human beings of ages between 23–56 years

Batch no.	Blood Group	SBP/DBP	BPR	BHCR	UCHI@37.5 °C
3073	O+	150/90	1.666	3.500	3.110
3074	A+	120/70	1.714	2.760	2.691
3078	B−	150/90	1.666	2.7292	2.709
3080	O+	150/90	1.666	2.9935	2.824
3082	A+	140/96	1.458	2.6759	2.640

**Figure 3:** Demonstrating the percentage variations of evolved gases (viz., N_2_ −m/z = 28, O_2_ −m/z = 32, CO_2_ −m/z = 44, Ar −m/z = 40, an unknown composite gas −m/z = 28.5) from the blood samples of four different healthy human beings and one guinea pig during the hyphenated technique at a blood temperature of 40 °C (104 F).

**Figure 4:** Mass spectrum of CO_2_ evolved as a function of both time and temperature in the blood samples of healthy subjects.^[^ ^1^ ^]^

It is crystal clear from Figure 4 that the possibilities of internal flow choking in the human being is higher than the animal (Guinea pig); under the same thermal loading condition as the BHCR of the dominant gas evolved in the animal is found to be consistently higher than in a human being. As a result, the LCHI is higher for the healthy male Guinea pig as dictated by the Equation (2). We have observed that the mass spectrum of N_2_ is found to be higher in the animal whereas in human beings CO_2_ is found to be higher.^[^ ^1^ ^]^ The BHCR of N_2_ is 1.4 and that of CO_2_ is 1.289. At this thermal loading condition, the animal artery gets choked only at a BPR of 1.8929 and the human artery gets an early choking at a BPR of 1.8257. Therefore, we concluded that the thermal tolerance level of the healthy Guinea pig is higher and the cardiovascular risk is lower than for a human being under identical conditions. On this rationale, increasing the thermal tolerance level in terms of BHCR of the human being is an important factor for reducing the risk of acute‐heart failure (AHF) due to the Covid‐19 or otherwise.

The article "Lopsided Blood‐Thinning Drug Increases the Risk of Internal Flow Choking Leading to Shock Wave Generation Causing Asymptomatic Cardiovascular Disease" was retracted in 2024. Reasons: unreliable results or conclusions; concerns about the data; concerns about the results or conclusions.

## 4 In Silico Methodology

In an effort to demonstrate the boundary layer induced Sanal flow choking followed by shock wave generation and transient pressure‐overshoot in an artery with divergence region, we have carried out single phase in silico studies with creeping inflow conditions (a case with gas embolism) using a validated flow solver.^[^ ^10^ ^]^ We could demonstrate the shock wave generation and pressure overshoot at the downstream region of an artery with a divergent region (see **Figure** **5**) leading to asymptomatic cardiovascular disease. The in silico result presented in Figure 5 clearly demonstrates the phenomenon of Sanal‐flow‐choking and shock waves generation at the subsonic inflow condition (creeping flow) leading to transient pressure‐overshoots (stroke) in the downstream region of an artery with a divergent port. During the in silico simulation we have also experienced streamtube flow choking^[^ ^39^, ^79^ ^]^ followed by the Sanal flow choking (see **Figure** **6**; Movie S2, Supporting Information). The Sanal flow choking^[^ ^1^ ^]^ and the streamtube flow choking^[^ ^39^, ^79^, ^81^ ^]^ are new theoretical concepts applicable to both the continuum and non‐continuum fluid flows. When the streamlines compressed, the pressure difference will be significant within the streamtube and the flow gets accelerated to a smaller area section of the streamtube for meeting the continuity condition, which leads to the Sanal flow choking and supersonic flow development at a critical‐total‐to‐static pressure ratio due to the convergent‐divergent (CD) shape of the streamtube. Herein, we provide the proof of the concept of fluid‐throat persuaded flow choking in the cardiovascular system. For establishing this concept authoritatively, we have presented an infallible closed‐form analytical model (see Equation (4a)) for predicting the 3D boundary layer displacement thickness (defined herein as 3D blockage factor) at the sonic‐fluid‐throat location where the slip length is zero, which will be a useful tool for the in vitro and in silico experiments in both the continuum and non‐continuum flows with due consideration of heat transfer effects (real‐world fluid flow effect). It corroborates that the phenomenon of Sanal flow choking is a paradigm shift in the diagnostic sciences of asymptomatic cardiovascular diseases. Therefore, development of a multi‐phase, multispecies, viscoelastic fluid‐structural interactive in silico model capturing the memory effect (stroke history) is a meaningful objective for predicting a priori the asymptomatic cardiovascular disease with credibility. Such an effort will be helpful for the diagnosis, prognosis, treatment, and prevention of the asymptomatic hemorrhage and acute heart failure of each and every subject with confidence.

The article "Lopsided Blood‐Thinning Drug Increases the Risk of Internal Flow Choking Leading to Shock Wave Generation Causing Asymptomatic Cardiovascular Disease" was retracted in 2024. Reasons: unreliable results or conclusions; concerns about the data; concerns about the results or conclusions.

**Figure 5:** In silico results show the Sanal‐flow‐choking and shock waves generation at the subsonic inflow condition (creeping flow) leading to the transient pressure overshoots (stroke) in the downstream region of an artery with divergent port as a result of the CD nozzle flow effect (a case with gas embolism). Also see Movie S2, Supporting Information.

**Figure 6:** Demonstrating the Sanal flow choking and streamtube flow choking condition in an idealized physical model of an artery with divergent port geometry at a critical pressure ratio with a creeping inflow condition.

## 5 Discussion

Although the diagnostic sciences have been advanced significantly during the last eight decades, until the dissemination of this article and connected articles,^[^ ^1^, ^10^, ^11^, ^12^, ^13^, ^14^, ^15^, ^79^, ^80^, ^81^, ^82^, ^83^ ^]^ the real occurrence of AHF remains poorly understood, largely for the reason that it was an under diagnosis condition.^[^ ^26^, ^27^, ^28^ ^]^ Now the real cause of an AHF comes to the foreground.^[^ ^1^, ^10^, ^11^, ^12^, ^13^, ^14^, ^15^, ^79^, ^80^, ^81^, ^82^, ^83^ ^]^ In patients with a recent history of the embolic stroke of undetermined source, dabigatran was found to be not superior to aspirin in preventing recurrent stroke.^[^ ^26^ ^]^ Based on a three clinical trials report, John W. McEvoy^[^ ^27^ ^]^ highlighted that aspirin for the primary prevention of cardiovascular disease has become increasingly hard to defend, however, the physician recommends that it is reasonable to continue aspirin with low‐dose for the subject, Mr. Evans, a 72‐year‐old man with blood pressure 130/72 with a diagnosis of external hemorrhoids. On the contrary, another physician, Sigrun Halvorsen^[^ ^27^ ^]^ recommends to the same subject, Mr. Evans, to stop taking aspirin because the absolute benefit associated with aspirin in this elderly man is small due to the increase in the risk of major bleeding. In brief, we recommended Mr. Evans should always maintain his systolic‐to‐diastolic BPR lower than LCHI through drugs or otherwise for an extended healthy life.^[^ ^1^ ^]^

Viscosity of blood is directly related to the number of red blood cells (hematocrit). Blood plasma has been considered a Newtonian fluid for decades but through experiments Brust et al.^[^ ^22^ ^]^ revealed that blood plasma has a pronounced viscoelastic behavior.^[^ ^23^ ^]^ Many studies have been carried out and reported worldwide on the variations of blood viscosity and seasonal changes on blood pressure (BP) causing several cardiovascular diseases.^[^ ^22^, ^23^, ^24^, ^25^, ^26^, ^27^, ^28^, ^29^, ^54^, ^55^, ^56^, ^57^, ^58^ ^]^ The viscoelastic material possesses a characteristic that can be referred to as a “memory effect,” (i.e., stress/stroke history herein). It means that the material response is not only determined by the current state of stress, but is also determined by all of the past stress histories.^[^ ^1^, ^59^ ^]^ Therefore, an accurate and a priori knowledge of the combined effect of rheology of biofluid and the thermoviscoelastic response of the vessels (the memory effect/stroke history) is inevitable for predicting acute heart failure using the fluid‐structural interactive code.^[^ ^10^ ^]^ All the findings reported and reviewed herein are complementary with the existing literature and clinical data on variations of blood viscosity and seasonal changes on blood pressure (BP) causing several cardiovascular diseases.^[^ ^60^, ^61^, ^62^, ^63^, ^64^, ^65^, ^66^, ^67^, ^68^, ^69^, ^70^, ^71^, ^72^, ^73^, ^74^, ^75^, ^76^, ^77^, ^78^, ^79^, ^80^, ^81^, ^82^, ^83^ ^]^

An internal flow choking in the cardiovascular system (CVS) leads to shock wave generation and pressure overshoot at various physical situations (see Figure 1) warranting memory effects (stroke history), which leads to a tear inside an artery (SCAD). When the inner layers of the artery separate from the outer layers, blood can pool in the area between the layers. The SCAD may slow blood flow through the artery to the heart, which makes the heart muscle weaken. Note that at the flow choking condition the shock wave generated by the individual nanoplasma at this physical situation is sufficient for creating an event of AHF. In certain situations a heart attack that is caused by hardening of the arteries (atherosclerosis) due to the memory effects (i.e., stroke history/pressure overshoots due to shock waves or shock diamonds) is also well known. In all these physical situations the effect due to the transient pressure‐overshoot was noticed.

The article "Lopsided Blood‐Thinning Drug Increases the Risk of Internal Flow Choking Leading to Shock Wave Generation Causing Asymptomatic Cardiovascular Disease" was retracted in 2024. Reasons: unreliable results or conclusions; concerns about the data; concerns about the results or conclusions.

The analytical models (Equations (1)–(5)), the in vitro and in silico results presented herein corroborated that a vaccination could reduce the risk of the asymptomatic hemorrhage and acute heart failure.^[^ ^1^, ^59^ ^]^ It could be achieved by increasing the BHCR of subjects in accordance with the BPR. In a nutshell, we have proved conclusively that the high‐heat capacity ratio (HCR) of blood reduces the risk of acute‐heart failure, which is an indisputable physical condition for prohibiting asymptomatic cardiovascular diseases (see Equations (1)–(5)).

We recognized that the internal flow choking, leading to shock wave generation and the transient pressure spike in a blood vessel, is the fundamental cause of asymptomatic hemorrhage and acute heart failure. Now the precipitating factor for the plaque rupture has come to the foreground. We concluded that biofluid choking (due to plaque induced blockage or due to vasospasm) and the Sanal‐flow‐choking (due to BLB) could occur anywhere in the circulatory circuit when BPR reaches LCHI. The BLB‐factor depends on the BHCR, flow Mach number, the biofluid viscosity, and turbulence, which could alter due to seasonal changes, variations in lipoprotein and other contributing factors. The greater the reduction in low‐density lipoprotein (LDL) cholesterol, the lower the risk of stroke. It is important to note that all the clinical findings are corroborative of the models presented herein for predicting the condition of prohibiting the asymptomatic cardiovascular diseases. The shock wave and cavitation could disrupt an atherosclerotic plaque or coronary artery wall. The cavitation is quite noisy and can be sufficiently violent to physically damage valves, arteries, and blood vessels.

All these studies lead to an authentic conclusion that the BHCR, the critical BPR, and memory effect (stroke history) are the key deciding factors for hemorrhagic stroke and acute heart failure. We concluded that high BHCR reduces the risk of asymptomatic hemorrhage and acute heart failure and that for a healthy‐life all human beings and animals with the high systolic‐to‐diastolic BPR (hypertension/hypotension subjects) invariably have to maintain high BHCR. In a nutshell, the discovery of the biofluid/Sanal‐flow‐choking is a paradigm shift in the diagnostic sciences of coronary artery disease (CAD) and peripheral artery disease (PAD).

Through closed‐form analytical models (see Equations (1)–(5)) we could correlate various controlling parameters of cardiovascular diseases, namely, BHCR, BPR, blood viscosity, and ejection fraction. It sheds light on finding solutions for decreasing the risk of asymptomatic hemorrhage and acute heart failure due to internal flow choking. In vitro studies are carried out on fresh blood samples of healthy subjects in the age group of 23–56 years from the southern part of the Indian union with diverse blood groups along with a healthy male Guinea pig of four weeks old.

An in vitro study shows that nitrogen (N_2_), oxygen (O_2_), carbon dioxide (CO_2_), and argon (Ar) gases are predominant in the fresh blood samples of healthy subjects at a temperature range of 37–40 °C (98.6–104 F), which enhances the chances of internal flow choking (with or without any coronary artery stent) leading to pressure‐overshoot and acute heart failure in Covid‐19 patients. We detected that CO_2_ gas generation is comparatively and persistently higher in healthy human beings than the healthy male Guinea pig. In vitro results show that BHCR of fresh blood samples are higher than those collected in three different Vacutainers of the same subjects. The thermal tolerance level of healthy Guinea‐pig is found to be greater and the cardiovascular risk is lesser than in the healthy human being. Analytical findings reveal (see Equation (5d)) that the relatively high and low blood viscosity values are cardiovascular risk factors. The fact is that when blood viscosity decreases Reynolds number increases, which contributes for increasing the turbulence level causing an early flow choking due to the enhanced BLB factor. An analytical model also reveals that at a constant ejection fraction, cardiovascular risk increases while decreasing the BHCR, reducing the DBP, and increasing the vessel blockage (plaque/boundary layer).

The article "Lopsided Blood‐Thinning Drug Increases the Risk of Internal Flow Choking Leading to Shock Wave Generation Causing Asymptomatic Cardiovascular Disease" was retracted in 2024. Reasons: unreliable results or conclusions; concerns about the data; concerns about the results or conclusions.

Using the compressible flow theory, Equations (1)–(5) are derived.^[^ ^10^, ^11^ ^]^ It is crystal clear from Equations (1), (5c), and (5d) that stenosis (an abnormal narrowing of the passage of a blood vessel, i.e., a decrease in hydraulic diameter of the blood vessel or a decrease in vessel cross‐sectional area) could increase the risk of internal flow choking. These equations (Equations (1), (5c), and (5d)) also tell us that a stent implant for increasing the hydraulic diameter could decrease the risk of internal flow choking but is not a permanent solution for reducing the risk of acute heart failure, without having proper control on the other influencing parameters highlighted herein (see Equations (1)–(5)). It is important to note that though all the existing percentage demarcations of the ejection fraction are meaningful for the diagnosis, these findings were not supported by any closed‐form analytical model for an authentic conclusion prior to the discovery of these analytical models. Note that until the dissemination of this article the desirable blood flow percentage or exact ejection fraction for healthy subjects for forecasting the risk of AHF was unknown to the scientific community. Note that Equations (1) and (5c) show the correlation of the ejection fraction in terms of the BFR of a normal heart with other controlling parameters (vessel geometry, fluid dynamics, and thermodynamic properties of blood/biofluid). These controlling parameters are explicitly highlighted in the mathematical models, which establish the condition for internal flow choking. More specifically, it is evident from the analytical models that the cardiovascular risk factor depends on the coupled effects of the ejection fraction, the vessel cross‐sectional area (*A*_local_), BHCR, DBP, Reynolds number, and the local velocity (*V*_local_). It is evident from these mathematical models that at a constant vessel cross sectional area and DBP decrease in BHCR and an increase in Reynolds number jointly or individually, increase the possibilities of internal flow choking. Apparently, (see Equation (5d)) an increase in kinematic viscosity increases the possibilities of internal flow choking. On the contrary, an increase in kinematic viscosity decreases the possibilities of internal flow choking by reducing the Reynolds number. It reveals that there is a safe range of blood viscosity for prohibiting the internal flow choking of each and every subject, which depends upon the coupled effects of the other controlling parameters (see Equations (1)–(5)) for the internal flow choking. Therefore, the dose of blood‐thinning drugs must be prescribed, subjected to the condition prescribed in the models. Based on the closed‐form analytical models (see Equations (2) and (2a)) we have reported conclusively that high BPR and low BHCR are risk factors for internal flow choking leading to asymptomatic hemorrhage and acute heart failure.

The article "Lopsided Blood‐Thinning Drug Increases the Risk of Internal Flow Choking Leading to Shock Wave Generation Causing Asymptomatic Cardiovascular Disease" was retracted in 2024. Reasons: unreliable results or conclusions; concerns about the data; concerns about the results or conclusions.

A randomized controlled in vitro study conducted using the Differential Scanning Calorimeter (DSC) – Perkin Elmer DSC 8000, reveals that blood is a compressible fluid. There are deviations found in the BHCR of fresh samples of blood collected in different Vacutainers for the same healthy subjects. The specific heat capacity (*C*_p_) of blood samples of healthy subjects (ages 22–58 years with different blood groups – ethical clearance is not required in India) taken from the EDTA and Lithium Heparin tubes were found to be 32.789% and 33.1594% lower, respectively, than the fresh samples of the same healthy subjects tested within 5 min of collection. It proves conclusively that drugs with anticoagulant properties reduce the BHCR and increase the risk of internal flow choking leading to the asymptomatic cardiovascular diseases. Through hyphenated techniques we could detect four known gases, namely, N_2_, O_2_, CO_2_, and Ar in the fresh blood samples of healthy subjects of human beings and an animal at 98.6–104° F. We observed that, carbon dioxide (CO_2_), the gas with the lowest HCR is relatively and consistently higher in the healthy males than the healthy male Guinea pig of four weeks old (see Figure 4). Note that HCR of CO_2_ is 1.289, therefore a subject with gas embolism, with CO_2_ as the dominant gas, the internal flow choking occurs at a BPR of 1.8257, which is the LCHI. It reveals that patients who are taking blood‐thinning medication must maintain their BPR always less than 1.8257, as dictated by Equation (2), for reducing the risk of asymptomatic cardiovascular diseases.

The article "Lopsided Blood‐Thinning Drug Increases the Risk of Internal Flow Choking Leading to Shock Wave Generation Causing Asymptomatic Cardiovascular Disease" was retracted in 2024. Reasons: unreliable results or conclusions; concerns about the data; concerns about the results or conclusions.

### 5.1 Clinical Perspectives: Competencies in Medical Knowledge

The BHCR, the critical BPR and memory effects (stroke history/internal flow choking history) are the major risk factors deciding the possibilities for the aneurysm, asymptomatic hemorrhage, and acute heart failure in all subjects. The analytical and the in vitro procedures described herein will play a key role in the future medical sciences for the prediction and negation of aneurysm, arrhythmia, hemorrhagic stroke, and myocardial infarction (MI) a priori, with or without symptoms of the plaque on the artery walls through new therapies, new drug discoveries, medical procedures, or diagnostics, namely, the estimation of the BHCR.

We presumed that thrombophilia, gas embolism, the blood glucose, and other property variations of blood could alter the BHCR of individual subjects, which could alter LCHI. We comprehended that in addition to the gene editing, within the framework of the pathophysiological constraints of individual subjects, the transfusion of blood with high HCR could negate the risk factor of the asymptomatic hemorrhage and acute heart failure in high‐risk subjects owing to the fact that it creates less chances of internal flow choking in the cardiovascular system.

### 5.2 Translational Outlook

Large randomized blood sample tests for BHCR, estimation along with the BPR measurement, adequately in all seasons in all blood groups, across the globe are needed for discovering new drugs capable of increasing the BHCR and/or decreasing the BPR in all seasons for reducing the risk of internal flow choking in all subjects. Note that the internal flow choking leads to acute myocardial infarction (MI) and asymptomatic strokes of various types. Therefore, BHCR of the Covid‐19 patients’ needs to be estimated for predicting the risk of a cardiovascular epidemic.

Randomized tests for thermo‐gravimetric, thermolysis, and speciation analyses of blood samples of all subjects, in all blood groups, in all geographical regions of the globe in all seasons are envisaged to check the thermal tolerance level and the cardiovascular risk of each and every subject.

This seminal review article opens a new avenue of research in biological and material sciences for accurately estimating memory effects for pinpointing the locations and conditions of plaque/artery rupture a priori through the analytical, in silico, in vitro, in situ or in vivo studies. The 3D printing model test, in situ or in vivo studies, are recommended for examining memory effects and the altered variations of the on‐site relaxation modulus of vessels. The in vitro estimation of the chemical and elemental species of each and every subject along with the blockage factor estimation are recommended for forecasting the risk of an early flow choking due to seasonal changes.

The article "Lopsided Blood‐Thinning Drug Increases the Risk of Internal Flow Choking Leading to Shock Wave Generation Causing Asymptomatic Cardiovascular Disease" was retracted in 2024. Reasons: unreliable results or conclusions; concerns about the data; concerns about the results or conclusions.

Animal models, without pain and mortality, are recommended for the parametric study of internal flow choking, aneurysm, arrhythmia, asymptomatic hemorrhage, and acute heart failure before proceeding for therapies in human being for lowering the risk of acute MI and improving clinical outcomes. The breakthrough concept of internal flow choking (biofluid/Sanal flow choking) phenomenon expedites the discovery of new diagnostic tools and treatments through our multidisciplinary collaboration.

### 5.3 Concluding Remarks

Mostly, in the cardiovascular system blood flow is considered as laminar. When taking blood thinning drugs, the whole blood viscosity reduces and as a consequence the Reynolds number rises and the laminar flow could be disordered and converted to turbulent. The flow turbulence enhances the deficit of energy in the type of friction, which increases the BLB in the vessels and generates heat and augments the internal energy affecting a reduction in BHCR, which is corroborated with in vitro results. Additionally, turbulence enhances the perfusion pressure essential to push the blood flow.

We concluded that a single anticoagulant drug capable of suppressing the turbulence level and enhancing the BHCR, or a companion medicine along with the traditional blood‐thinning medications is predestined for meeting the conflicting requirements (i.e., decrease viscosity and turbulence simultaneously) of all the subjects for reducing the risk of asymptomatic hemorrhage and acute heart failure. In high risk subjects (i.e., BPR is very close to the LCHI) a slight oscillation in the BPR predisposes to the choking and the unchoking phenomena, which could lead to arrhythmia and memory effect. In a nutshell, we have proved conclusively that the high‐BHCR reduces the risk of internal flow choking as dictated by Equation (2), which is an indisputable physical condition, without any ex vivo or in vivo model support, for prohibiting asymptomatic cardiovascular diseases. We concluded that internal flow choking occurs in an artery with and without stent. We also concluded that for a healthy‐life all subjects with high BPR inevitably have high BHCR. This review article sheds light for exploring new avenues in biological science for discovering new blood‐thinning drugs for reducing the risk of internal flow choking causing asymptomatic hemorrhage and acute heart failure.^[^ ^1^ ^]^ We concluded that the cardiovascular treatment should be targeted based on BPR, instead of blood pressure levels alone, in chronic heart failure patients.^[^ ^40^, ^41^ ^]^

Briefly, we concluded that the risk of internal flow choking heading to asymptomatic hemorrhage and acute heart failure could be decreased by concurrently reducing blood viscosity and turbulence by enhancing the BHCR or reducing the BPR. This manuscript discloses new insights into the cardiovascular epidemic of the 21st century and the associated disease process that allow researchers to design drugs through nanotechnology with a proper chemical composition worldwide for increasing the BHCR and for reducing the risk of a cardiovascular epidemic due to the Covid‐19 pandemic. Note that when the pressure of the nanofluid increases, the average mean free path decreases and thus, the Knudsen number reduces leading to a no‐slip boundary condition with a compressible viscous flow effect. The Sanal‐flow‐choking is a compressible viscous flow effect, which is established as the flow choking caused by the BLB at the creeping inflow condition at a critical pressure ratio. The Sanal‐flow‐choking is an undesirable phenomenon, which could cause asymptomatic stroke and/or acute heart failure in Covid‐19 patients. The sporadic internal flow choking, due to significant fluctuations in BPR, heading to transient pressure‐overshoots created throughout a life‐span in the cardiovascular system, creates vessel walls which are stiffer due to memory effects (stroke history). Such physical situations in any of the viscoelastic vessels are prone to rupture in the subsequent internal flow choking and shock wave development. We concluded that the risk of internal flow choking leading to asymptomatic hemorrhage and acute heart failure could be reduced by concurrently reducing blood viscosity and turbulence by enhancing the BHCR (i.e., increasing the thermal tolerance level) or decreasing the BPR. In light of the recent guidance of the European Society of Cardiology,^[^ ^41^ ^]^ this manuscript is submitted to the global community for discovering a brilliant chemical formula urgently for increasing the thermal tolerance level of all human beings worldwide after due consideration of the pathophysiological constraints of individual subjects for clinical trials for prohibiting the cardiovascular epidemic in Covid‐19 patients and also for the general categories through proper medical management.

The article "Lopsided Blood‐Thinning Drug Increases the Risk of Internal Flow Choking Leading to Shock Wave Generation Causing Asymptomatic Cardiovascular Disease" was retracted in 2024. Reasons: unreliable results or conclusions; concerns about the data; concerns about the results or conclusions.

The scientific objective of this study and review was to discover the correlation between the thermal tolerance level in terms of BHCR, the BPR, blood viscosity, ejection fraction, and the cardiovascular risk leading to asymptomatic hemorrhage and acute heart failure, which we could achieve herein. We concluded that designing a precise blood thinning regimen is vital for attaining the desired therapeutic efficacy and negating undesirable flow choking leading to acute‐heart failure. The uneven usage of blood‐thinning drugs enhances the risk of the internal flow choking owing to the enhanced BLB due to turbulence. For a healthy‐life all subjects with high‐BPR inevitably have high‐BHCR for reducing the risk of the internal flow choking (biofluid/Sanal‐flow‐choking) triggering acute heart failure due to shock wave generation. We corroborated that, the acute heart failure is a transient episode and not an illness.^[^ ^1^, ^8^, ^9^ ^]^

Briefly, we could establish herein that at the creeping inflow condition there are possibilities of the generation of shock waves followed by transient pressure‐overshoot in the cardiovascular system having convergent‐divergent (CD) duct (due to plaque deposit or BLB) flow region immediately after the internal flow choking (biofluid choking and/or Sanal flow choking). The discovery of the Sanal flow choking phenomena calls for a continuous ambulatory blood pressure (BP)^[^ ^71^ ^]^ and thermal level monitoring in high risk patients in the diagnosis and preventive management of asymptomatic cardiovascular diseases.^[^ ^71^, ^72^, ^73^, ^74^, ^75^, ^76^, ^77^, ^78^ ^]^ Continuous blood pressure and thermal level measurement could be done in a more pragmatic way by using a wearable BP monitor with a temperature sensor in the modern form of a wristwatch. Analytical methods such as machine learning could definitely enhance accuracy and advance daily wearable device‐based diagnoses. Of late (2020) Amrith Mariappan et al.^[^ ^84^ ^]^ reported that the silicon powder obtained from the recycling of space debris could be used for producing feigned soil for fostering pharmaceutical flora in the International Space Station (ISS) to discover scarce‐drugs for increasing the BHCR for high‐endurance health care management. M. D. Delp et al.^[^ ^85^ ^]^ highlighted that Apollo lunar astronauts exhibit higher cardiovascular disease mortality. It is known that cardiovascular risk is higher in astronauts/cosmonauts but the fundamental cause of such risk was unknown to medical science^[^ ^79^, ^84^, ^85^, ^86^, ^87^ ^]^ until the dissemination of this article and our connected articles.^[^ ^1^, ^10^, ^11^, ^12^, ^13^, ^14^, ^15^, ^79^ ^]^ The beauty and novelty of the internal choking phenomenon, discovered in the cardiovascular system and nanoscale system, reviewed herein is that the causes and effects of the Sanal flow choking in cardiovascular system satisfy all the clinical findings world‐wide (catalogued and non‐catalogued) pertaining to the risk factors of asymptomatic cardiovascular diseases reported over the centuries.

The article "Lopsided Blood‐Thinning Drug Increases the Risk of Internal Flow Choking Leading to Shock Wave Generation Causing Asymptomatic Cardiovascular Disease" was retracted in 2024. Reasons: unreliable results or conclusions; concerns about the data; concerns about the results or conclusions.

## 6 Significance Statement

Acute heart failure (AHF) is the biggest killer world‐wide. Through analytical, in vitro, and in silico studies the authors demonstrated that a disproportionate blood thinning treatment increases the threat of asymptomatic cardiovascular disease (CVD). For maintaining a healthy life all subjects (human being/animal) with high‐BPR inevitably have blood with high‐heat capacity ratio for reducing the risk of internal flow choking and associated asymptomatic CVD. Drugs capable of enhancing the thermal tolerance could diminish the cardiovascular‐risk in all subjects including the Covid‐19 patients. The authors found out that at a critical BPR the Sanal flow choking occurs in the cardiovascular‐system with sudden expansion/divergence/vasospasm/bifurcation regions leading to the generation of shock waves and a transient sharp pressure‐spike causing asymptomatic‐hemorrhage (AH) and acute heart failure (AHF). This review article sheds light for exploring new avenues in biological science for discovering new blood‐thinning drugs for reducing the risk of internal flow choking causing AH and AHF in the Covid‐19 patients and also in the general category.

## Conflict of Interest

The authors declare no conflict of interest.

## Author Contributions

V.R.S.K.: Conceptualization, analytical modeling, manuscript drafting; S.K.C.: In vitro conceptualization, manuscript editing; P.K.R.: In vitro conceptualization, manuscript editing; R.S.B.: In vitro and data generation; N.C.: In vitro, in silico, and project support, V.S.: Modeling and simulation support, A.S.: In silico simulation support, C.O.: Resources.

## Supporting information

Supporting Information

Supplemental Video 1
